This article has been retracted.

# Exploration of the Cultivation Path of Medical Students' Politico-Ideological and Humanistic Quality Based on Deep Learning

**DOI:** 10.1155/2022/5766675

**Published:** 2022-06-28

**Authors:** Sainan Xue, Shuang Li

**Affiliations:** College of Nursing, Inner Mongolia Medical University, Hohhot, Inner Mongolia Autonomous Region 010059, China

## Abstract

Medical talent development has its own characteristics, which means that political-ideological education in medical colleges must establish a development model that reflects these characteristics. In a methodological sense, research on the development of politico-ideological education in medical colleges should adhere to the coordinated development of politico-ideological education in medical colleges, which follows the requirements of the current situation and the three laws of politico-ideological education in medical colleges, namely, the requirements of the law of politico-ideological education, the law of teaching and educating people, and the law of study. In practice, in view of the practical contradictions in the politico-ideological work of medical colleges and universities at the present stage, explore the collaborative education mechanism of medical colleges and universities, constantly enrich the ways and methods of politico-ideological work in medical colleges and universities, improve the affinity, pertinence, and effectiveness of politico-ideological education, and constantly open up a new situation of politico-ideological education in colleges and universities. This work offers a path exploration approach based on deep learning for cultivating the political-ideological, and humanistic qualities of medical students' curriculum, and the model's performance is proven by simulation trials.

## 1. Introduction

The Communist Party of China has always attached great importance to politico-ideological work. The discipline of politico-ideological education was established in the early 1980s, and the politico-ideological work in colleges and universities began to be highly valued in the late 1980s [1]. The discipline of politico-ideological education has developed rapidly at this stage, and the discipline system, content, media, and means of politico-ideological education are also constantly improving. At the same time, under the background of the rapid development of economy and society, the rapid change of science and technology, and the continuous improvement of the level of opening to the outside world in the period of social transformation, there are many challenges and problems in the continuous development and self-improvement of politico-ideological education in colleges and universities [2], including the challenge of the development concept of western universities, the challenge of hostile forces at home and abroad, the challenge of multiple ideologies and values, and the challenge of new media. The unique history, culture, and national conditions determine that we must take our own path of higher education development [3]. Do a good job of running socialist colleges and universities with Chinese characteristics and putting them in a strong position to follow the party's leadership. Fully implementing the party's education policy, policy, and line, continuously strengthening and improving politico-ideological education, always adhering to the correct direction of educating people, and comprehensively improving the politico-ideological work of colleges and universities are all critical [4]. The significance and ways of humanistic quality and politico-ideological education in colleges and universities are shown in Figure 1.

It is of great significance to fully implement the party's education policy, policy, and line, continuously strengthen and improve politico-ideological education, always adhere to the correct direction of educating people, and comprehensively improve the politico-ideological work of colleges and universities [5]. It is conducive to solving the current politico-ideological education dilemma and enhancing the effectiveness of politico-ideological education in medical schools. It is conducive to the issue of improving the ideological and moral quality of medical students and implementing the concept of synergy in the politico-ideological education of medical schools [6]. Through the organic integration of curriculum thinking and political science courses, which can better penetrate the notion of educational thought, the organic integration of medical professional teaching and political-ideological education teaching can be realized. Teaching through practice bases, such as university hospital internships and community clinics, cultivates the spirit of medicine, enhances the apprehension of the meaning of life, helps motivate the learning of professional skills, and facilitates the cultivation of new medical talents with both virtues and talents [7]. The research on the collaborative development of politico-ideological education in medical schools under the pattern of “Big Thinking and Politics” is conducive to building a smooth communication channel in education and teaching, bringing into play the affinity of politico-ideological work, enhancing the effectiveness of education, and facilitating the integration of the links and communication among the constituent elements and departments in the current education system, so as to bring into play the proper functions of each subsystem.

Compared with the traditional politico-ideological education mode, the “great politico-ideological” education mode has its own characteristics [8]. First of all, the education mode under the “great politico-ideological” pattern has the universality of personnel participation. In terms of participants, the education mode under the “great politico-ideological” pattern is not limited to full-time teachers of politico-ideological theory courses but requires the teaching staff of the whole school to participate in the politico-ideological work of college students. Secondly, the educational mode under the pattern of “great thought and politics” has the extensive use of time and space. Colleges and universities should shoulder the task of educating people all the time from entering the school to graduation and in all educational links. In talent training, education, and teaching, we should adhere to the principle of education first and moral education first and pay attention to and implement the infiltration method of politico-ideological education [9]. Thirdly, due to the pertinence and openness of the content system, the politico-ideological education in colleges and universities has vitality. It must keep up with the pace of the times and always adhere to being close to reality and life [10]. The politico-ideological education should be targeted and the content selection of politico-ideological education should be open. Politico-ideological education should face the world and the future, absorb the advanced achievements of human civilization to the greatest extent, release the attraction and appeal of politico-ideological education to the greatest extent, and improve the affinity of politico-ideological education. Finally, the platform makes use of the complementarity of virtual reality [11]. In terms of educational methods and means, based on the characteristics of the network era, integrate the real platform and virtual platform, and strive to truly promote the cultivation of morality in the complementary advantages of multiple platforms.

The arrangements of the paper are as follows: Section 2 discusses the related work.  Section 3 describes the design of application model.  Section 4 examines the experiments and results; section 5 concludes the article.

## 2. Related Work

### 2.1. Research Status of Humanistic Quality Education for Medical Students

Medical students' humanistic education needs to go through two stages: the classroom learning stage and the clinical practice stage. Similar to the current situation the biomedical model is still dominant in clinics, China's medical education has not gotten rid of the traditional biomedical education model. In the classroom learning stage, whether it is basic medical courses or clinical courses, teachers only pay attention to the explanation of medical knowledge [12]. Ignoring the explanation of humanistic knowledge combined with clinical practice leads medical students to know little about doctor-patient communication skills and the complex doctor-patient relationships. Clinical practice is an important period for medical students to learn. It is a key stage to combine the theoretical knowledge of classroom learning with clinical practice. However, at present, the humanistic education of medical students in clinical practice has not been paid attention to [13]. The current situation of humanistic education for medical students is shown in Figure 2.

Most of the teachers in clinical teaching units have been used to the disease-centered biomedical model. They believe that medical knowledge and technology are the most important. Students with solid clinical knowledge and skills can be competent for clinical work. Most of the clinical teaching teachers are frontline clinical doctors. They are nervous and do not have enough time to lead students to communicate with patients on the spot [14]. However, students' work stays on the writing of medical documents. Some teaching teachers have insufficient humanistic knowledge reserves and cannot play an exemplary role for students. Some teachers are afraid of medical disputes and dare not let medical students contact patients, which deprives medical students of the opportunity to combine the learned humanistic knowledge with clinical practice and cannot effectively transform it into clinical ability. All of these hinder the improvement of medical students' humanistic quality and make students have the idea of emphasizing technology over humanities [15]. Teachers are the key factor in the cultivation of the humanistic quality of medical students. At present, the number of teachers in medical colleges in China is insufficient and the structure of teachers is unreasonable. Teachers of general medical courses graduated from medical colleges and universities, with good medical professional knowledge, but lack humanistic knowledge [16]. Humanities teachers graduated from nonmedical colleges and lack a comprehensive and systematic understanding of medical knowledge. Teachers act in their own way and lack communication and exchange, so they cannot organically combine the medical knowledge and humanistic knowledge learned by students. The frequent occurrence of doctor-patient disputes, especially violent medical injuries, has a certain negative impact on the humanistic education of medical students [17]. On the one hand, it makes them lack confidence and even fear about the career they want to engage in the future, which leads some medical students to switch to other careers after leaving school [18]. On the other hand, in order to avoid the occurrence of medical disputes, some clinical practice units dare not let interns operate or communicate with patients, which deprives them of a great opportunity to integrate theory with practice.

### 2.2. Research Status of Politico-Ideological Education for Medical Students

In fact, in clinical work, we often find that some patients are resistant to interns and unwilling to cooperate with their diagnosis and treatment activities, so they cannot master doctor-patient communication skills well [19]. The lack of doctor-patient communication skills of medical students is easy to cause contradictions with patients in their contact with patients and leads to doctor-patient disputes. This will create a vicious cycle that is not helpful to the development of a positive doctor-patient relationship. Medical colleges and universities, like the majority of colleges and universities, struggle with issues such as ideological imbalance between teachers and students, a single teaching paradigm, and a lack of an overarching idea of politico-ideological education [20]. At the same time, the problems of politico-ideological education in medical colleges still have their particularity, the lack of personality in politico-ideological education, and so on. The above problems pose a great challenge to the effectiveness of politico-ideological education in medical colleges. It is urgent to change the development mode of politico-ideological education in medical colleges and take coordinated development as the methodological guidance [21]. The coordinated development of politico-ideological education in medical colleges and universities refers to taking the concept of coordinated development as the methodological guidance of the action of politico-ideological education in medical colleges and universities in order to achieve the goal of politico-ideological education [22]. The structure of politico-ideological education in medical colleges is shown in Figure 3.

The coordinated development of politico-ideological education in medical colleges can learn from various educational media, educational subjects, and other favorable factors and operate in a coordinated and orderly manner [23]. Thus, the functions of each part can be brought into full play, and the goal of politico-ideological education in medical colleges can be optimally and effectively realized. Professional course teachers and politico-ideological theory teachers should cooperate to educate people and do well the politico-ideological work in medical colleges and universities [9]. We should follow the law of politico-ideological work, the law of teaching and educating people, and the law of students' growth and constantly improve the ability and level of politico-ideological work. To make good use of the classroom as the main channel, the theory course of politico-ideological education should be strengthened in improvement, enhance the affinity and pertinence of politico-ideological education, and meet the needs and expectations of student's growth and development [24]. Educators are the first to receive an education. Only under the guidance of educators with noble moral quality and keeping pace with the times, can they smoothly interact with the educated in the process of education, so as to improve students' ideological and moral quality. The success of this interaction ultimately depends on the teacher as the leader of education [25].

### 2.3. Research Status of Deep Learning

How to transfer the input data from the original space to the high-dimensional space, which can distinguish two types of complicated sample data without requiring any implicit mapping kernel function [26], is a problem worth considering. A good way to overcome this problem is to utilize a deep neural network to map the samples from input space to feature space, which will improve the classification effect. Generally speaking, for a given number of training samples, if they lack other prior knowledge, people prefer to use a small number of calculation units to establish the compact expression of the objective function in order to obtain better generalization ability. Deep learning takes the original form of data as the input of the algorithm [27]. The original data is abstracted layer by layer as the final feature representation required by its own task and finally ends with the mapping from the feature to the task target. In particular, experience has proved that the two-stage strategy composed of unsupervised pretraining and supervised tuning is not only effective for overcoming the training difficulties of deep networks but also endows deep networks with superior feature learning ability. Then, many new depth structures were established. Meanwhile, at last year's international top conference on computer vision and pattern recognition, researchers announced the end of the ImageNet challenge [28]. Even though it has only been around for eight years, it has accomplished incredible things. Machine learning has advanced in the disciplines of computer vision, speech recognition, and natural language processing, while the outcomes of picture categorization and target identification have made significant advances.

Among them, the key is that the neural network has ushered in its spring again after a long cold winter. Although deep learning can automatically obtain features of different scales from simple to abstract when using the extracted features for classification or recognition, a deep neural network uses the feature of the last hidden layer for classification, that is, using the feature of a single scale for classification [29]. This is because, in the deep neural network, a layer is connected with its front and rear adjacent layers, that is, it can only receive input from the adjacent previous layer.

## 3. Design of Application Model

Based on deep learning, this paper focuses on the kernel mapping structure and spanning structure model of the deep neural network, in order to effectively solve the shortcomings of the original method, improve the performance and generalization ability of the deep neural network, and finally promote the improvement and development of deep neural network model. This research plays a positive role in promoting the development of deep neural networks, especially multilayer perceptron and convolutional neural network models. Combined with the research focus of this paper, some representative works in multicore learning and cross-connected convolution neural networks are introduced in detail. Among them, the research of multicore learning is mainly divided into the research of learning methods of multicore learning and the research of training methods of multicore learning. The three representative models of cross-connected convolutional neural networks are fast track network, residual network, and densely connected network. When the compound nucleus is applied to the task of gene function classification, the classification accuracy is higher than that of a single nucleus. The mathematical expression is as follows:

(1) $$\begin{array}{c} \begin{array}{c} K_{\text{comb}}=K_{1}\left(x_{1}+x_{2}\right)+K_{2}\left(x_{1}+x_{2}\right),\\ K_{\text{comb}}=K_{1}\left(x_{1}+x_{2}\right)\cdot K_{2}\left(x_{1}+x_{2}\right). \end{array} \end{array}$$

Then, the combination coefficient is directly calculated through a heuristic process, and its mathematical expression is as follows:

(2) $$\begin{array}{c} A\left(K,K_{t}\right)=\frac{{\langle K,K_{t}\rangle }_{F}}{\sqrt{{\langle K,K\rangle }_{F}{\langle K_{t},K_{t}\rangle }_{F}}}. \end{array}$$

The weight in the classification function leads to the combination kernel function with worse performance. Therefore, the kernel matrix is obtained first.

(3) $$\begin{array}{c} K^{c}=K-\frac{1}{n}1\cdot 1^{T}\cdot K-\frac{1}{n}K\cdot 1\cdot 1^{T}+\frac{1}{n^{2}}\left(1^{T}\cdot K\cdot 1\right)\cdot 1\cdot 1^{T}. \end{array}$$

Then, calculate the combination coefficient as shown below, and a more reasonable combination kernel function can be obtained.

(4) $$\begin{array}{c} \theta_{m}=\frac{A\left(K_{m}^{c},K_{t}^{c}\right)}{\sum_{i=1}^{M}\;A\left(K_{i}^{c},K_{t}^{c}\right)}. \end{array}$$

The optimization method also expresses the composite kernel function as a nonnegative linear combination of a set of basis kernels. The difference is that it calculates the combination coefficient through some optimization criterion.

(5) max∑m=1M θmyTKmys.t.∑m=1M ∑i=1M θmθiKm,KiF=c θ∈R+M.

By solving the programming problem represented by the above formula, the combination coefficient can be obtained. Moreover, the optimization method can also express the composite kernel function as the nonlinear combination of the base kernel. The mathematical expression of its objective function is as follows:

(6) $$\begin{array}{c} \begin{array}{c} \underset{W,b,\theta }{\min}\;\;\frac{1}{2}W^{T}W+\underset{l}{\sum }\;L\left(y^{l},f\left(x^{l}\right)\right)+r\left(\theta \right)\\ \text{ s}.\text{t}.\;\theta \in R_{+}^{M} \end{array}. \end{array}$$

Kernel functions can have a variety of forms, commonly used for the following mathematical expressions:

(7) $$\begin{array}{c} K_{\text{comb}}\left(x_{i},x_{j}\right)={\left(d_{0}+\overset{M}{\underset{m=1}{\sum }}\;\theta_{m}x_{i}^{T}x_{j}\right)}^{q}. \end{array}$$

The depth method is to stack multiple basis kernels in depth to obtain the composite kernel function and then use some criteria to solve the parameters. The structural block diagram of the composite kernel function of the depth method is shown in Figure 4.

The optimization problem of multilayer and multicore learning of *j*-layer can be expressed as

(8) $$\begin{array}{c} \underset{K\in K^{\left(j\right)}}{\min}\;\underset{f\in H_{K}}{\min}\;\lambda {\left\|f\right\|}_{H_{K}}+\overset{N}{\underset{l=1}{\sum }}\;L\left(y^{l}f\left(x^{l}\right)\right). \end{array}$$

Specifically, the mathematical of the decision function can be expressed as

(9) $$\begin{array}{c} K^{\left(2\right)}=\left\{K^{\left(2\right)}\left(x_{i},x_{j};\theta \right)=\exp\left(\overset{M}{\underset{m=1}{\sum }}\;\theta_{m}K_{m}^{\left(1\right)}\left(x_{i},x_{j}\right)\right)\right\}. \end{array}$$

At this time, the mathematical expression of the objective function is

(10) $$\begin{array}{c} \underset{K\in K^{\left(2\right)}}{\min}\;\underset{f\in H_{K}}{\min}\;\frac{1}{2}{\left\|f\right\|}_{H_{K}}^{2}+C\overset{N}{\underset{l=1}{\sum }}\;\max\left(0,1-y^{l}f\left(x^{l}\right)\right)+\overset{M}{\underset{m=1}{\sum }}\;\theta_{m}. \end{array}$$

Firstly, the base core is selected, and then, the selected base core is combined in a linear or nonlinear way to obtain the composite core. However, research shows that the composite kernel generated by multicore learning is not always better than the base kernel, one possible reason is that the network structure of multicore learning is shallow and has certain limitations, which is not enough to express relatively complex composite kernel functions through the linear or nonlinear combination of base kernels. Most of the current multicore learning methods convert the problem to dual space and use a two-step method to solve the parameters. This will cause misunderstanding among readers to a certain extent. For solving the kernel learning method, we must convert it to dual space for the solution. The cross-layer connection structure of the residual network is shown in Figure 5.

The traditional deep neural network only allows the structure connected by adjacent layers, which limits its integration of multiscale features for classification or recognition. In the fast-track network, information can flow across layers directly behind layers without obstacles, and its mathematical expression is as follows:

(11) $$\begin{array}{c} y=H\left(x,W_{H}\right)\circ T\left(x,W_{T}\right)+x\circ C\left(x,W_{C}\right). \end{array}$$

By multiplying element by element, the fast tracklayer can be simplified to

(12) $$\begin{array}{c} y=H\left(x,W_{H}\right)\circ T\left(x,W_{T}\right)+x\circ \left(1-T\left(x,W_{H}\right)\right). \end{array}$$

Another treatment is to change the dimension of the ordinary layer first and then stack the fast track layer. Based on these two processes, a similar fast tracklayer can be constructed by using the idea of shared weight and receptive field in a convolutional neural network. Once convergence begins, degradation problems may also occur. The degradation problem is that as the depth increases, the accuracy quickly reaches saturation and then degenerates rapidly. Unexpectedly, this degradation is not caused by overfitting, because increasing the number of layers will lead to a higher error rate. The introduction of identity transformation can make the adjustment of network. Parameters more effective, i.e., the mapping is more sensitive to output change after the introduction of residual. In terms of back-propagation, identity mapping allows for direct propagation and the addition of the error term to the front layer, removing gradient reduction and explosion issues. In short, residuals allow you to remove the same main part while highlighting minor differences. According to research on residual networks, even networks with hundreds of layers can be trained reliably and successfully provided cross-layer connections are added between levels. Broadly speaking, a dense network refers to a convolutional neural network containing one or more dense modules, as shown in Figure 6.

This control of growth rate cannot only reduce the parameters of the dense network but also ensure the performance of the dense network. However, dense networks simply splice features of different scales, which may lead to feature redundancy. In addition, the dense network consumes a lot of memory during training. The usual approach is to design a cross-connect structure carefully for a given task. This approach usually achieves good results but does not provide people with the difference between the results of different cross-connect methods. To sum up, this paper proposes a deep neural mapping support vector machine model. The model uses a deep neural network to explicitly represent the kernel mapping and maps the input from the original space to the feature space. In fact, kernel mapping is an explicit function represented by a deep neural network.

## 4. Experiments and Results

In order to accurately understand the current situation of the implementation of curriculum politico-ideological education, a questionnaire survey was conducted on the teaching front-line teachers of the teaching part of 8 medical colleges in Shandong and some students in freshman, sophomore, and junior grades, and field visits were conducted to investigate the politico-ideological classroom of relevant schools. The teaching records of politico-ideological education were included in the scope of this study, so as to master the specific implementation of curriculum politico-ideological education such as students' cognitive status and teachers' cognitive status. Starting with the current situation of curriculum politico-ideological education, this paper deeply explores and analyzes the bottlenecks and reasons encountered in the implementation process, puts forward reasonable solutions for the implementation of curriculum politico-ideological education in the classroom, and puts forward measures to improve the quality of curriculum politico-ideological education, so as to integrate teaching with politico-ideological education and improve the ideological and moral level of medical students. The current situation of politico-ideological integration is shown in Table 1 and Figure 7.

The results show that in the implementation of curriculum thought and politics, the integration of physical education in sophomore is the best, followed by the freshman, and the integration of junior is slightly worse. On the one hand, it may be related to the learning pressure of students. Compared with freshmen and sophomores, junior students are facing great pressure of graduation. The focus of learning is on the subjects of cultural courses, which requires a lot of time to study and review cultural courses. On the other hand, some politico-ideological courses may be replaced by other teachers, resulting in the reduction of students' politico-ideological courses. At the same time, in order to serve other courses, teachers only complete teaching tasks in class, only pay attention to the teaching of skills and ignore the guidance of values, which makes it difficult to implement curriculum politico-ideological education in the third grade. In contrast, freshmen and sophomores face less pressure. Sophomores have adapted to the school environment, have a certain sports foundation, and have stronger autonomy in choosing learning content, so it is easier to implement curriculum thought and politics. Through the investigation, it is found that in terms of the ways to receive politico-ideological education, students believe that politico-ideological course is the main way to carry out politico-ideological education, followed by the infiltration in various disciplines, indicating two problems: one is that high school students lack ideological education at present, and the other is that the school does not pay attention to carrying out ideological education. The statistics of politico-ideological elements in the end part are shown in Table 2 and Figure 8.

From the results of teachers' questionnaire statistics, first, in terms of teachers' cognition, teachers believe that the current way for students to receive ideological education is through the penetration of various disciplines. Secondly, most teachers affirmed the suitability and necessity of curriculum politico-ideological infiltration into the classroom and said that they would implement it in the follow-up classroom, but on the whole, teachers' understanding of curriculum politico-ideological is not enough.

## 5. Conclusion

People benefit from political-ideological education. The work of being a man is difficult, and the ideological work of being a man is even more difficult. In general, political-ideological education integrates individual differences with society's mainstream values. Individuals have subjective initiative, and there are still some distinctions among them. Medical colleges and universities should be transformed into model places of stability and unity in order to cultivate a pleasant and welcoming environment. The politico-ideological education in medical colleges and universities should proceed from reality and integrate theory with practice. Based on this, this paper proposes a path exploration method for the cultivation of politico-ideological, and humanistic quality of medical students' curriculum based on deep learning, and the effectiveness of the model is verified by simulation experiments.

The research on the coordinated development of politico-ideological education in medical colleges is a research focusing on practice and application. In the future, we should continue to think about how to do a good job in the politico-ideological education in medical colleges and improve the affinity and pertinence of the politico-ideological education in medical colleges. Politico-ideological educators should have strong theoretical literacy and actively make use of the collaborative resources of Politico-ideological education with the characteristics and advantages of medical colleges. Finally, we should constantly improve our comprehensive ability to obtain and process information and be good at using new media. Other fields' mature theoretical and practical experience have been incorporated by the subject of political-ideological education. At home and abroad, dialectically treat and absorb ideological culture, science, and technology, and the discipline of politico-ideological education is expected to grow by leaps and bounds only via continual learning.

## Figures and Tables

**Figure 1:** The significance and ways of humanistic quality and politico-ideological education in colleges and universities.

**Figure 2:** The current situation of humanistic education for medical students.

**Figure 3:** The structure of politico-ideological education in medical colleges.

**Figure 4:** Diagram of the composite kernel function of the depth method.

**Figure 5:** The cross-layer connection structure of the residual network.

**Figure 6:** The convolutional neural network containing one or more dense modules.

**Figure 7:** The current situation of politico-ideological integration of the curriculum.

**Figure 8:** The statistics of politico-ideological elements in the end part.

**Table 1:** The current situation of politico-ideological integration of the curriculum.

	Freshman	Sophomore	Junior
Integration into curriculum thought and politics	11	14	9
Not integrated into the curriculum of politico-ideological education	21	18	23

**Table 2:** The statistics of politico-ideological elements in the end part.

Category	Relaxation activities	Mutual evaluation	Class summary	Job arrangement	Interaction
Numbers	22	34	342	21	35
Percentage	28.21%	43.59%	41.05%	26.92%	44.87%

## Data Availability

The datasets used during the current study are available from the corresponding author on reasonable request.
